# Infiltration and Significance of CD103+CD8+ T Cells in Gastrointestinal Adenocarcinoma

This article has been retracted.

**DOI:** 10.1155/2022/7469041

**Published:** 2022-09-09

**Authors:** Weisu Cai, Haitao Wang

**Affiliations:** ^1^Emergency Department, Changzhou Cancer Hospital Affiliated to Suzhou University, Changzhou 213000, China; ^2^Gastrointestinal Surgery, The Third Affiliated Hospital of Suzhou University, Changzhou 213000, China

## Abstract

Immunohistochemical staining is a common technique to study tissue morphology and in situ protein expression. With the rise of immunotherapy, more and more markers in the tumor microenvironment have been discovered. In this paper, the multiplex immunofluorescence staining method was used to stain paraffin sections of 35 cases of gastric adenocarcinoma tissue and 35 cases of colorectal adenocarcinoma tissue and its adjacent tissue. The infiltration of CD8+ T cells and CD103+CD8+ T cells in the slices was detected by using the slice scanner to form the map and CaseViewer2.0 software analysis. The experimental results in this paper showed that compared with adjacent tissues, the infiltration degree of CD8+ T cells in gastric adenocarcinoma tissue was significantly lower (*Z* = 2.244, *P* = 0.025, *P* < 0.05), and the infiltration degree of cells was significantly lower (*Z* = 2.785, *P* = 0.005, *P* < 0.05). In gastric adenocarcinoma tissue, the infiltration of CD8+ T cells was correlated with the tumor diameter of gastric adenocarcinoma (*P* = 0.002). There was a statistically significant difference. The degree of CD103+CD8+ T cell infiltration was related to the survival of patients with gastric adenocarcinoma (*P* = 0.002) and the degree of tumor differentiation (*P* = 0.004). The infiltration of CD103+CD8+ T cells in gastric cancer tissue and colorectal cancer tissue is related to the survival of patients. CD103+CD8+ T cells are thought to play a role in the prognosis of gastric adenocarcinoma and colorectal adenocarcinoma. Experiments have shown that the more the CD103+CD8+ T cells, the better the prognosis of gastric adenocarcinoma and colorectal adenocarcinoma, so the prognosis of gastric adenocarcinoma and colorectal adenocarcinoma can be improved by increasing CD103+CD8+ T cells.

## 1. Introduction

Gastric cancer not only will cause damage to the digestive system but also may metastasize, affecting the liver, kidney, and respiratory functions. Gastric adenocarcinoma is a malignant tumor that occurs in the stomach, and the nature of this malignant tumor is called adenocarcinoma. Adenocarcinoma is a kind of cancer in medical terms, cancer is a kind of malignant tumor, and malignant tumor mainly includes two categories: carcinoma and sarcoma. In China, the rate of colorectal cancer has risen dramatically in recent years. The most frequent malignant tumor in the world, with substantial morbidity and mortality, is the gastrointestinal tumor. According to the American Cancer Society's 2018 World Cancer Statistics, stomach cancer has the fifth highest incidence and the third highest fatality rate in the world. In addition, China has a high incidence of stomach cancer. Gastric cancer was the third most common cancer in 2018, with a 10.6 percent incidence rate and a 13.6 percent fatality rate. In 2018, the global incidence of colorectal cancer was 6.1 percent, putting it in the fourth place, and the fatality rate was 9.2 percent, putting it in the second place. Colorectal cancer has become more common in China in recent years.

Gastric tumors can be prevented by eradicating Helicobacter pylori, recommending good living habits, and regular gastroscopy screening for high-risk groups for early diagnosis and early treatment. At present, the etiology of gastrointestinal tumors is still unclear. The high incidence of gastric cancer may be related to geographical factors, dietary habits, Helicobacter pylori, precancerous lesions, genetics, and other factors. In recent years, high-risk factors related to colorectal cancer have gradually been recognized, such as high-fat, high-animal protein diet, long-term lack of fresh vegetables, and crude fiber foods. Genetic susceptibility also plays an important role in the incidence of colorectal cancer.

The innovations of this paper are as follows: (1) the theoretical knowledge of gastrointestinal adenocarcinoma tissues and CD103+CD8+ T cells is introduced, and the flexible neural tree algorithm is used to analyze the infiltration of CD103+CD8+ T cells in gastrointestinal adenocarcinoma tissues and meaning. (2) The flexible neural tree algorithm and DNA microarray technology were described, and it was found through experiments that CD103+CD8+ T cell exposure affects the development of gastrointestinal adenocarcinoma.

## 2. Related Work

Gastrointestinal disease, as the name suggests, refers to functional abnormalities or inflammation of the stomach and intestines, including ulcers, tumors, and other diseases. Usually, chronic gastrointestinal diseases do not necessarily occur at the same time and can simply manifest as chronic gastritis, gastric ulcer, and gastric tumor. With the improvement of people's living standards these years, the diet has become more and more diversified, which has led to the emergence of many gastrointestinal diseases. Zeichner et al. found that over the past 20 years, there has also been a radical change in the understanding of the mechanisms of cancer metastasis, with treatments in oncology now being incorporated into the clinical care of patients in the United States. While diagnostic tests for metastatic GA (mGA) may improve patients' ability to prevent disease, the gap is still large, but it is about the same cost as other drugs [1]. Saito et al. discovered a rare example of a collision tumor with primary jejunal adenocarcinoma and gastrointestinal stromal tumor (GIST). Furthermore, this patient also suffered from gastrointestinal and duodenal distension. He was diagnosed with primary adenocarcinoma. The scholar has been emphasizing the patient's symptoms and has not given a solution [2]. Imtiyaz et al. found that hypoxia-inducible factor can regulate energy cell homeostasis and improve tumorigenesis. However, no relationship has been found, and in order to fully characterize cellular adaptation to hypoxia, the different functions of the two must be compared. But the scholar did not express how to conduct the experiment [3]. Hirota et al. found that cell survival is determined by the tumor necrosis factor receptor (TNFR) and Fas (CD95) can signal apoptosis through an established pathway. In the adult nervous system, Fas also causes apoptosis. However, during the development of the nervous system, Fas can also make neurite outgrowth and branch outgrowth rapidly, and the process induced by Fas has not been explored. But Hirota et al. did not specify the role of the cell [4]. Peters et al. found that tumors can evade immune-mediated destruction, and inhibition of lymphocyte infiltration or effector function can be combined to achieve this goal, but new methods must be investigated to overcome the difficulties and thereby enhance the tumor-killing ability of tumor-reactive lymphocytes. If you want to improve its working efficiency, you can combine it with interleukin cytokines. But the scholar did not explain how to improve its work efficiency [5].

## 3. Influence of the Degree of Infiltration of CD103+CD8+ T Cells in Gastrointestinal Adenocarcinoma

### 3.1. The Development Trend of Gastrointestinal Adenocarcinoma

A tumor can be thought of as an immunocompromised disease, where the failure of immune recognition results in malignant cells growing into tumors. There are three distinct steps in tumorigenesis: the inefficient clearance of early transformed cells. Cancers evade or alter the host's immune response in various ways to ensure its development and survival [6]. Innate immune recognition molecules are all proteins encoded by germline genes, but some molecules such as the classical complement pathway recognition molecule C1q, the alternative pathway recognition molecule C3, and the peptidoglycan recognition protein have not been classified, and it still being discovered. Innate immune recognition molecules can also be functionally divided into humoral proteins circulating in plasma, endocytic receptors expressed on the cell surface, and signaling receptors on the cell surface or in cells. The innate immune system includes a series of cells and related mechanisms that can defend against foreign infection in a nonspecific manner. Cells of the innate immune system recognize and act on pathogens nonspecifically.

Cancer cells reproduce very fast, and normal cells cannot get sufficient nutrients and oxygen. Cancer cells will directly release toxins, affecting organs and reducing organ function. If you always have indigestion and no appetite, you should go to the hospital for examination in time. You must not ignore some abnormalities in digestive function. Various diseases have evolved as a result of human birth, and humans have begun to suffer from the harm and invasion of these diseases [7, 8]. Cancer is the most serious threat to human health among them [9]. When a patient is diagnosed with cancer in medicine, they are usually in the middle or late stages of the disease, which results in a high mortality rate for cancer patients.  Figure 1 depicts the increase rate of stomach cancer patients from 2012 to 2021.

As shown in Figure 1, explore the molecular mechanism of gastric cancer etiology, and find biomarkers for diagnosis and prognosis; it is imperative to study treatment goals [10]. The molecular mechanism refers to the influence of cellular molecular substances involved in or produced in the process of cell metabolism on the regulation, growth, and survival of cells, including macromolecular substances and small molecular substances.

New cases of gastric cancer account for more than 40% of new cases in the world every year, and the mortality rate ranks second. This is a major disease that seriously endangers health. The proportion of gastric cancer patients in China is very high, and the 5-year survival rate after comprehensive treatment with surgery as the mainstay is also very low [11]. The mortality and survival rates from 2016 to 2018 are shown in Figure 2.

As shown in Figure 2, the occurrence of gastric cancer is caused by a combination of factors. The most common causes include Helicobacter pylori infection, precancerous lesions, genetic factors, and environmental and dietary factors. The etiology of gastric cancer is complex, including genetic factors, environmental factors, and other aspects. In order to expand the treatment methods of gastric cancer, improve the survival of gastric cancer patients, explore the molecular mechanism of gastric cancer etiology, and find biomarkers for diagnosis and prognosis; more and more scholars conduct research on therapeutic targets [12]. Existing chronic inflammation, atrophic gastritis, atrophic gastritis with intestinal metaplasia, dysplasia, and other diseases, under the action of Helicobacter pylori infection, unhealthy diet, and bad environment, gradually transform to gastric cancer.

### 3.2. DNA Microarray Technology

The detection of human genes by DNA microarrays and the guidance of clinical treatment have become a new hotspot in today's scientific field. The emergence of microarrays provides a new tool for the detection of gene expression of chemotherapeutic drugs. DNA microarray is also known as DNA array or DNA chip, and the more popular name is gene chip. It is a special glass slide coated with DNA microarray. Thousands or tens of thousands of nucleic acid probes are installed on an area of several square centimeters. After one test, a large amount of gene sequence-related information can be provided. Fluorescence intensity information for gene discovery is obtained by fluorescence microscopy or laser detection of the Gundam chip, and the information is obtained using image processing and analysis software. Genetic factors include genes. Specifically, it is the nature and shape of the organism, such as size, height, and color. “Traits” are superficial phenomena that people perceive, and their recurrence has some inherent reason. The discovery value of the genetic factor is usually expressed as the logarithmic ratio of the two fluorescence intensities expressed as

(1) $$\begin{array}{c} \text{gen}\_\text{expression}=\log\frac{\text{Int}\left(\text{Cb}5\right)}{\text{Int}\left(\text{Cb}5\right)}. \end{array}$$

The *m*∗*n* data matrix formed by the found values of *m* genes determined in *n* experiments is the DNA microarray data of

(2) $$\begin{array}{c} M=\left[\begin{array}{ccc} a_{11} & a_{12} & a_{1n}\\ a_{21} & a_{22} & a_{2n}\\ a_{m1} & a_{m2} & a_{nm} \end{array}\right]. \end{array}$$

Column vector *a*_*nm*_ represents the expression level of *m* genes in the *j*th experiment.

Microarray data analysis is a sequence analysis method for high-throughput genotyping and expression analysis. Microarrays can generate high-quality data and enable academic and research institutions to rapidly complete large-scale *P* studies. In order to facilitate the subsequent analysis of the data, each element in the microarray data needs to be within the same range. The process of converting all data to the same dimension is called data normalization [13]. Let *a*_*ij*_ and *a* be used to represent the original expression value and the normalized value of gene *i* on the *j*th sample, respectively. Normalization is a way of simplifying the calculation; that is, the dimensional expression is transformed into a dimensionless expression and becomes a scalar. This method is often used in various calculations. The two most commonly used microarray data normalization methods are described below:

(3) $$\begin{array}{c} a_{ij}=\frac{\left(a_{ij}-a_{\min}\right)}{a_{\max}-a_{\min}}. \end{array}$$

Among them, *a*_min_ and *a*_max_ represent the minimum and maximum values of gene *i* in all samples, respectively. Another standardization method is to standardize by formula (3), so that the variance of each gene is 1 and the mean value is 0. The specific calculation is as follows:

(4) $$\begin{array}{c} a_{ij}=\frac{\left(a_{ij}-\overset{-}{a_{i}}\right)}{\delta },\\ \overset{-}{a_{i}}=\frac{1}{n}\overset{n}{\underset{j=1}{\sum }}a_{ij},\\ \delta =\sqrt{\frac{1}{n-1}\overset{n}{\underset{j=1}{\sum }}\left(a_{ij}-\overset{-}{a_{i}}\right)}. \end{array}$$

Among them, $\overset{-}{a_{i}}$ and *δ* represent the mean and standard deviation of gene *i* in all samples, respectively.

Tumor is a cell in the local tissue that loses its normal growth regulation at the gene level under the action of a variety of carcinogenic causes, resulting in its clonal abnormal proliferation and the formation of a new organism. Cell proliferation is the basis for the growth, development, reproduction, and inheritance of organisms. Cloning broadly refers to making an exact replica of a particular organism. In biology, it refers to the selective cloning of a DNA sequence, cell, or individual. The ratio of the sum of squares between genes to the sum of squares within a class is proposed as

(5) $$\begin{array}{c} \text{BW}\left(j\right)=\frac{\sum_{i}\sum_{k}\left(b_{i}-k\right){\left(a_{kj}-a_{j}\right)}^{2}}{b_{i}}. \end{array}$$

Among them, (*b*_*i*_ − *k*) is a discriminant function, which is used to determine to which category the current sample belongs. The higher the ratio of BW(*j*), the more significant the difference in gene expression of gene *j* between samples in different categories and the smaller the difference in gene expression within the same category. Based on this, the ratio of all genes was calculated, and the *P* genes with the highest ratio were selected [14].

A flexible neural tree (FNT) is a new type of tree model, similar to a neural network. In this paper, tree structure coding is adopted, and the neural tree structure is optimized by a multiexpression programming algorithm. The flexible neural tree model is constructed by simple predefinition, which can solve the problem of high structure dependence of the artificial neural network. The flexible neural tree model not only can avoid complicated calculation and circuit connection but also has high real-time recognition rate and low root mean square error. The flexible neural tree model is composed of two types of instruction sets: functional instruction set (denoted by *F*) and terminal instruction set (denoted by *T*) [15]. The functional instruction set is composed of nonleaf nodes in the flexible neural tree, and the terminal nodes are composed of input features. The model of FNT can be expressed as

(6) $$\begin{array}{c} S=F\cup T=\left\{+2,+3,\cdots ,+N\right\}\cup \left\{a_{1},a_{2},\cdots ,a_{n}\right\}. \end{array}$$

{*a*_1_, *a*_2_, ⋯, *a*_*n*_} represents a leaf node without any parameters, which is actually an input feature variable.

In a neural network, there is a functional relationship between the input and output of the hidden layer and output layer nodes, and this function is called the excitation function. In the process of creating the tree structure of flexible neural tree, the Gaussian distribution function is often used as the excitation function of nonleaf nodes. Instructions are randomly selected from the instruction set, each node in the neural network accepts the input value and passes the input value to the next layer, and the input node will directly pass the input attribute value to the next layer (hidden layer or output layer). In a neural network, there is a functional relationship between the input and output of the hidden layer and output layer nodes, and this function is called the excitation function. The excitation function of nonleaf nodes is

(7) $$\begin{array}{c} f\left(a,a_{i},b_{i}\right)=e^{-1/2}. \end{array}$$

The formula for calculating the total excitation result of neuron + *i* is

(8) $$\begin{array}{c} {\text{net}}_{i}=\overset{i}{\underset{j=1}{\sum }}w_{j}\times a_{j}, \end{array}$$

where *w*_*j*_ represents each input of the node; then, the output of the node is shown in

(9) $$\begin{array}{c} {\text{out}}_{i}=f\left({\text{net}}_{i},a_{i},b_{i}\right). \end{array}$$

It is very important to select an appropriate fitness function in FNT, not only to be able to describe the quality of a flexible neural tree but also to reflect the error between the actual output and the expected output. Several commonly used fitness functions are introduced below [16]. The fitness function satisfies the conditions of continuous differentiability, and the only requirement is that the nonnegative result that can be compared can be calculated for the input. The absolute error and calculation formula are shown in

(10) $$\begin{array}{c} \text{fitness}\left(i\right)=\overset{n}{\underset{j=1}{\sum }}\left|b_{0}^{j}-b^{j}\right|. \end{array}$$

The calculation formula of the mean square error is

(11) $$\begin{array}{c} \text{fitness}\left(i\right)=\frac{1}{N}\overset{n}{\underset{j=1}{\sum }}{\left(b_{0}^{j}-b^{j}\right)}^{2}. \end{array}$$

The root mean square error (RMSE) calculation formula is shown in

(12) $$\begin{array}{c} \text{fitness}\left(i\right)=\sqrt{\frac{1}{N}\overset{n}{\underset{j=1}{\sum }}{\left(b_{0}^{j}-b^{j}\right)}^{2}}. \end{array}$$

There are two types of learning in flexible neural trees: generation-based learning (GBL) and elite learning (EL). For flexible neural trees, generation-based learning is the most common learning approach [17]. The goal of elite learning is to employ the greatest program available as a starting point. Formula (13) depicts the PIPE execution process:

(13) $$\begin{array}{c} P_{\left(d,w\right)}\left(I\right)=\frac{PT}{l}. \end{array}$$

### 3.3. Characteristics of Memory T Cells and Their Role in Tumor Immunity

Memory T cells (TM) are human immune cells. The third line of defense of human immunity is divided into two parts: one is humoral immunity and the other is cellular immunity. After T cells divide and differentiate, memory T cells and effector T cells are formed, respectively. The development and formation process of memory T cells are not fully understood at present, and it is still uncertain whether memory T cells evolve from effector T cells or develop from another pathway. There are currently three different differentiation models for the formation of CD8+ memory T cells [18].

In the first model, CD8+ T cells differentiate according to a linear pathway. That is, all CD8+ T cells differentiate at the final stage, and a few cells continue to differentiate during the systolic phase, becoming memory T cells with long-term survival and proliferation ability.

In the second model, activated CD8+ T cells will slowly differentiate, which will cause death after exertion. CD8+ T cells generally refer to cytotoxic T lymphocytes. Cytotoxic T lymphocytes (CTL), a subset of leukocytes, are a kind of specific T cells that secrete various cytokines to participate in immune function. It has a killing effect on certain viruses, tumor cells, and other antigenic substances and constitutes an important defense line of the body's antivirus and antitumor immunity with natural killer cells. As the immune response progresses, the death signal is not fully detected or is not reversible, allowing surviving T cells to become memory T cells.

In the third model, effector T cells and memory T cells are differentiated from different precursor cells. In conclusion, it is still unclear which way memory T cells differentiate, and further research is needed to clarify. Memory T cells are shown in Figure 3.

As shown in Figure 3, tissue-resident memory T cells are a special subset of tumor-infiltrating lymphocytes (TILs) that can reside in tissues indefinitely and can rapidly respond to their cognate antigens. In recent years, another important type of memory T cells, tissue-resident memory T cells (TRM), has been discovered. TRMs do not express CCR7 and CD62L but highly express CD69 and/or CD103 and do not participate in the systemic circulation. The main function of tissue-resident memory T cells is to provide local protection against reinfection, but they are detrimental in organ transplantation. TRMs enable rapid and critical immune responses to localized pathogens without the need for recruitment of peripheral blood T cells.

### 3.4. Clinical Significance and Function of Memory T Cells

It is like a home that cannot function if it is full of garbage; a cell becomes unhealthy if it does not throw away the garbage it produces, but the cell can break it down to make energy. This process of TEM is called autophagy. The proliferative capacities of TEM and TCM were also different at different stages of infection. In the early stage of pathogens invading the body, TEM rapidly proliferates and plays a protective role against infection at the first time. TCM is the abbreviation of central memory T cell, which is a long-term memory T cell generated by naive T cells after antigen activation and can home to lymph nodes to receive antigen restimulation, while in the terminal stage of infection, TCM plays a leading role in immune defense, for example, in pneumonia caused by type B parainfluenza virus. T cell subsets with low or no expression of CD62L played a role, while T cell subsets with high expression of CD62L play a role.

TRM is an independent subgroup different from TEM and TCM. It is widely distributed in a variety of peripheral organs, including the brain, lung, gastrointestinal tract, urinary tract, female reproductive tract, and skin. Recent studies have shown that in lymphoid organs, TRM are also found in the thymus, lymph nodes, and spleen. When a certain part of the body is attacked by pathogens, the specific TRM in the tissue directly produces a rapid and specific immune response. For example, when the brain tissue is attacked by a virus, it can kill the virus, play a role in immune surveillance of the body, and can also initiate an immune response and play a role in resisting the virus.

### 3.5. The Relationship between Memory T Cells and Tumor Immunotherapy

A large number of studies have found that memory CD8+ T cells have a high frequency of self-renewal and can enable experimental mice to obtain antitumor protection. This provides strong evidence for the antitumor effect of memory T cells. Some scholars have proposed that memory T cells can be activated at lower concentrations of antigen to exert antitumor immunity. In vitro experiments have confirmed that memory T cells can release a large number of effective cytokines (INF-*γ*, IL-4, etc.) after activation to improve the tumor-killing effect.

Different subtypes of memory T cells play different roles in antitumor immunity. Some scholars have found CD8+ TEM infiltration in tumor tissue by immunohistochemical staining of rectal cancer living specimens and proved that the degree of infiltration is closely related to the tumor stage. Research findings also proved that CD8+ TEM mediates tumor immune response. After injecting TEM and TCM into experimental mice, the results show that a small part of TCM can maintain its phenotype, while TEM rapidly enters the terminal stage of differentiation and then undergoes apoptosis. This proves that TCM can also induce tumor immune function, and its killing ability in vivo is better than that of TEM. Scholars have also confirmed that TCM has a stronger tumor-killing effect than TEM.

### 3.6. The Relationship between the Infiltration Degree of CD8+ T Cells in Gastrointestinal Adenocarcinoma and the Clinicopathological Characteristics of Patients

The optimal cut-off value of X-tile software to analyze CD8+ T quantity in gastric adenocarcinoma tissue is 7.88 (cells/HPF). According to the best cut-off value, the samples are grouped. Different clinicopathological features were analyzed by Fisher's exact test, and the results are shown in Table 1.

As shown in Table 1, the degree of infiltration of CD8+ T cells is inseparable from the tumor diameter factor of gastric adenocarcinoma. The tumor diameter of gastric adenocarcinoma patients with highly infiltrated CD8+ T cells ≤ 5 cm is significantly higher than that of the high tumor diameter of 5 cm. The five-year survival period of patients after surgery also affects the degree of CD8+ T cell infiltration, and the proportion of patients with postoperative survival of 5 years is significantly higher than that of patients with survival period of ≤5 years.

### 3.7. The Relationship between the Infiltration Degree of CD8+ T Cells in Colorectal Adenocarcinoma and the Clinicopathological Characteristics of Patients

The relationship between the two results is shown in Table 2.

As shown in Table 2, according to the best cut-off value, the samples are grouped; CD8+ T quantity in colorectal adenocarcinoma tissue ≤ 7.2 (cells/HPF) is defined as the low-invasive group, the CD8+ T amount of 7.2 (cells/HPF) was defined as the high infiltration group.

### 3.8. The Relationship between the Infiltration Degree of CD8+ T Cells and Tumor Types

The optimal cut-off value of CD8+ T quantity in the total samples of gastric adenocarcinoma and colorectal adenocarcinoma analyzed by X-tile software was 8.76 (cells/HPF). The samples were grouped by the best cut-off value. The results are shown in Table 3.

As shown in Table 3, the degree of infiltration of CD8+ T cells was not significantly different between gastric adenocarcinoma and colorectal adenocarcinoma.

## 4. Experiment and Analysis of the Degree of Infiltration of CD8+ T Cells in Gastrointestinal Adenocarcinoma

### 4.1. Sample Selection and Case Data

In preliminary experiments, it was found that the fluorescence staining effect of CD103+CD8+ in undifferentiated cancers in gastric cancer and colorectal cancer is poor, and its expression is very low or even not expressed, while squamous cell carcinoma and carcinoid in gastric cancer and colorectal cancer are relatively rare. In gastric adenocarcinoma and colorectal adenocarcinoma, the CD103+CD8+ fluorescent staining effect is ideal, which is helpful for the identification of marked cells, and the pathological types are more common in clinic.

During the follow-up, two patients were found to be lost to follow-up, and a total of 70 cases were enrolled. Among these cases, 35 cases of gastric adenocarcinoma and 35 cases of colorectal adenocarcinoma were diagnosed by pathology, as shown in Table 4.

As shown in Table 4, in this study, 70 cases of paraffin tissue specimens of surgically resected tissue were selected in this study, and the adjacent tissue (surgical margin tissue) was taken as the control. Postoperative pathology confirmed gastric adenocarcinoma or colorectal adenocarcinoma. All cases had complete clinical data, and they did not receive chemotherapy, radiotherapy, or other antitumor adjuvant therapy before surgery.

### 4.2. The Relationship between the Degree of Infiltration of CD8+ T Cells in Gastrointestinal Adenocarcinoma and the Prognosis of Patients

The effect of CD8+ T cell infiltration on the survival of gastric adenocarcinoma patients is shown in Figure 4.

As shown in Figure 4, early gastric cancer is mainly controlled by diet, such as avoiding long-term consumption of pickled, smoked, and other foods, consuming low-salt and low-fat diet, and eating more vegetables, fruits, and other fiber-rich foods for prevention. Early gastric cancer has no specific symptoms. Patients and doctors pay little attention to the number and length of symptoms. If people investigate carefully, a series of clues will become clear. If the cancerous part blocks the pylorus, early satiety (including fullness and abdominal distention) occurs. In particular in the case of a regressed tumor with less curvature of the stomach, it may be reminiscent of a peptic ulcer. Stomach heart cancer can block the outlet of the esophagus, causing loss of appetite. A hard-shaped stomach on an X-ray, or a hypertrophic stomach lining in the esophagus on a CT scan, can be confused with esophageal cancer or painless disease even after careful study.

### 4.3. Multiplex Immunofluorescence Staining Experimental Steps

1. For sectioning, place the selected tissue paraffin block on the freezing table for half an hour, and after trimming, cut it into 3-5 *μ*m paraffin strips with a microtome
2. Take out the section, remove the secondary antibody, and immerse and wash the section in PBS for 3 times for 5 minutes each time
3. Add DAPI staining solution dropwise to each slice, about 10 *μ*l per slice, completely cover the tissue, spread the slices in a water-added incubation box, and incubate at room temperature for 10 minutes
4. Immerse and wash the stained sections in PBS for 3 times, lasting 5 minutes each time
5. Drop the antifluorescence quenching sealing solution on the surface of each sliced tissue, and seal the slices with a coverslip

Both CD8 and CD103 staining were localized on the cell membrane, the nucleus was blue, and the cell membrane was stained with a red ring, which was expressed as CD8+ cells.

The results of multiple immunofluorescence staining of gastrointestinal adenocarcinoma are shown in Figures 5–7.

In Figure 5, cell nucleus staining (DAPI) (Figure 5(a)), DAPI+CD8 staining (Figure 5(b)), DAPI+CD103 staining (Figure 5(c)), and DAPI+CD8+CD103 staining (Figure 5(a)) are shown; yellow arrows are CD8+ T cells, and white arrows are CD103+CD8+ T cells.

In Figure 6, cell nucleus staining (DAPI) (Figure 6(a)), DAPI+CD8 staining (Figure 6(b)), DAPI+CD103 staining (Figure 6(c)), and DAPI+CD8+CD103 staining (Figure 6(d)) are shown; yellow arrows are CD8+ T cells, and white arrows are CD103+CD8+ T cells.

In Figure 7, adenocarcinoma or esophageal tumor is suggested to be of gastric origin. Recent evidence is that this cancer may arise from a cylindrical abnormality in the lower end of the esophagus (ballet esophagus). Loss of weight and strength is often caused by dietary restrictions, for which patients come to the hospital. Massive serum or bleeding is rare.

Gastric adenocarcinoma, colorectal adenocarcinoma, and CD103+CD8+ T cells infiltrating these adjacent tissues are shown in Figures 8–10.

As shown in Figures 8–10, cells both infiltrated gastrointestinal cancer tissue and paracancerous tissue, colorectal adenocarcinoma tissue, and paracancerous tissue. Compared with adjacent tissues, the proportion of positive T cells did not change significantly.

In addition, the sample size can be increased, and the experiment can be repeated many times to verify the reliability of the conclusions. At the same time, it can be further studied under more clinical case characteristics, such as tumor marker values, erythrocyte sedimentation rate, the number of tumor-positive lymph nodes in postoperative specimens, and the proportion of positive lymph nodes in total lymph nodes. The clinical significance of CD103+CD8+T cell infiltration in a tumor was further studied through experiments.

## 5. Discussion

Tumor-related data in humans show that in different tumors, including early-stage non-small-cell lung cancer, lung squamous cell carcinoma, and high-grade serous epithelial ovarian cancer, tumors with TRM phenotype cell infiltration are related to better overall survival rate. Tumor immunotherapy using an immunization route that can generate TRM may have advantages in generating antitumor immunity. As a population of tumor-specific TRM cells, CD103+CD8+ T cells are generated similar to persistent infection, and tumor-specific CD103+CD8+ T cells are exposed to their cognate antigens for a long time. Because these CD103+CD8+ T cells can survive with the main tumor for years, they may play a function in tumor transformation control. Therapeutic stimulation of tumor-specific CD103+CD8+ T cells, as well as other resident cells, can boost local antitumor immune responses, aid tumor cell clearance, and lessen systemic side effects. To make therapeutic use of this feature, some viral vectors can be envisaged to efficiently generate localized CD103+CD8+ T cells by a limited number of peripheral tumor-specific effector cells. Alternatively, the antitumor activity of endogenous or therapeutic CD103+CD8+ T can be enhanced by blocking the junction with specific inhibitors.

## 6. Conclusions

Tumor immunity is an important means of treating tumors, and memory T cells play a unique and important role in antitumor immunity, which can improve the durability and effectiveness of treatment. Methods for improving the responsiveness of memory T cells and methods for enabling memory T cells to reach tumor sites and kill tumor cells are scientific issues that require further research. Moreover, if the subset of memory T cells is different, the surface markers, clinical characteristics, and antitumor effects are also different. Therefore, for different tumors, which memory T cells are necessary to induce is also the direction of future research.

## Figures and Tables

**Figure 1:** Growth rate of gastric cancer patients from 2012 to 2021.

**Figure 2:** Mortality and survival (2016-2018).

**Figure 3:** Memory T cells.

**Figure 4:** The effect of CD8+ T cell infiltration on the survival of gastric adenocarcinoma patients.

**Figure 5:** Fluorescent staining of gastric adenocarcinoma tissue.

**Figure 6:** Fluorescent staining of colon cancer tissue.

**Figure 7:** Fluorescent staining of rectal cancer tissue.

**Figure 8:** Fluorescence staining results of gastric adenocarcinoma tissue.

**Figure 9:** Fluorescent staining results of colon adenocarcinoma tissue.

**Figure 10:** The fluorescent staining results of rectal adenocarcinoma tissue.

**Table 1:** The relationship between the infiltration of CD8+ T cells in gastric adenocarcinoma and the clinicopathological characteristics of patients.

Clinicopathological features	Total	The number of CD8+ T cells ≤ 7.88 (cells/HPF)	The number of CD8+ T cells was 7.88 (cells/HPF)
Male	38	10	28
Female	7	5	2
Tumor diameter > 5 cm	19	5	14
Tumor diameter ≤ 5 cm	26	6	20

**Table 2:** The relationship between the infiltration of CD8+ T cells in colorectal adenocarcinoma and the clinicopathological characteristics of the patients.

Clinicopathological features	Total	CD8+ T quantity ≤ 7.2 (cells/HPF)	The number of CD8+ T cells was 7.2 (cells/HPF)
Male	29	7	22
Female	26	8	18
Tumor diameter > 5 cm	19	7	12
Tumor diameter ≤ 5 cm	26	10	16

**Table 3:** Relationship between infiltration of CD8+ T cells and tumor types.

Clinicopathological features	Total	CD8+ T quantity ≤ 8.76 (cells/HPF)	The number of CD8+ T cells was 8.76 (cells/HPF)
Gastric adenocarcinoma	30	10	20
Colorectal adenocarcinoma	25	9	16
Difference	5	1	4

**Table 4:** Cases of gastric adenocarcinoma and colorectal adenocarcinoma.

Clinicopathological features	Number of gastric adenocarcinoma cases (number)	Number of colorectal adenocarcinoma cases (number)
Male	15	10
Female	5	8
≤60 years old	3	8
>60 years old	12	9

## Data Availability

No data were used to support this study.
